# The Correlation between Serum Sclerostin Level and Arterial Stiffness in Peritoneal Dialysis Patients

This article has been retracted.

**DOI:** 10.1155/2022/4247782

**Published:** 2022-08-10

**Authors:** Fang Liu, Hongbin Ma, Yongfeng Ma, Wei Zhou, Chenlu Wang, Yongli Xiong

**Affiliations:** ^1^Department of Kidney Diseases, Shexian Hospital of Traditional Chinese Medicine, Huangshan, Hebei, China; ^2^Medical Department, Shexian Hospital of Traditional Chinese Medicine, Huangshan, Hebei, China; ^3^Laboratory, Shexian Hospital of Traditional Chinese Medicine, Huangshan, Hebei, China; ^4^Department of Radiology, Shexian Hospital of Traditional Chinese Medicine, Huangshan, Hebei, China; ^5^Department of Function, Shexian Hospital of Traditional Chinese Medicine, Huangshan, Hebei, China; ^6^Department of Science and Teach, Shexian Hospital of Traditional Chinese Medicine, Huangshan, Hebei, China

## Abstract

**Objective:**

To study the correlation between serum sclerostin (SO) and arterial stiffness in peritoneal dialysis (PD) patients.

**Methods:**

The study included 50 Parkinson's disease (PD) patients on continuous ambulatory peritoneal dialysis (CAPD) for more than 6 months at the nephrology department of our hospital. Without regard for age, the eligible patients were assigned to a low PWV group and a high PWV group with brachial-ankle pulse wave velocity (Ba PWV) of 1400 cm/s as the cutoff value. Patient characteristics such as age, gender, height, weight, BMI, smoking history, dialysis age, systolic blood pressure (SBP), diastolic blood pressure (DBP), urea clearance index (Kt/V), residual renal function (RRF), and diabetes mellitus (DM) were analyzed. Biochemical indices for analysis include hemoglobin (Hb), albumin (ALB), total cholesterol (TC), urea nitrogen (BUN), creatinine (CREA), triglyceride (TG), uric acid (UA), parathyroid hormone (PTH), blood phosphorus(P), fasting blood glucose (GLU), corrective calcium (Ca), calcium-phosphorus product, low-density lipoprotein (LDL-C), high-density lipoprotein (HDL-C), SO, and arterial stiffness.

**Results:**

There were 9 males and 16 females in the low PWV group and 12 males and 13 females in the high PWV group. Statistical significance was absent in patient characteristics despite more males in the high PWV group (*P*=0.055). The low PWV group had significantly lower mean age, SBP, SO, and PWV level, fewer diabetic patients, and higher CREA than the control group. Analysis of PWV-related factors showed that PWV was positively correlated with age, P, Ca, GLU, SBP, PTH, and SO while negatively correlated with CREA. Multiple stepwise regression analysis showed that age, SO, and SBP demonstrated great potential to predict PWV (*P* < 0.05).

**Conclusion:**

The degree of vascular sclerosis is highly correlated with SO level in Parkinson's disease patients, which might provide a theoretical basis for the evaluation of cardiovascular illness in Parkinson's disease patients. High serum sclerostin level is a risk factor for deteriorated arterial stiffness. Given the limited sample size, the relevant results require further validation by expanding the sample size.

## 1. Introduction

The mortality rate of end-stage renal disease (ESRD) accounts for about 20% of all renal diseases, posing a great threat to the patients [1, 2]. The clinical efficacy of the two commonly used continuous renal replacement therapies (CRRTs), peritoneal dialysis (PD) and hemodialysis (HD), is similar [3]. PD patients are predisposed to complications such as calcium-phosphate metabolic disorders and bone lesions. Despite previous evidence on the varying magnitude of correlation between SO level and arterial stiffness, discrepancies result in compromised research outcomes [4, 5]. Research [6] showed that with prolonged dialysis, about 61.6% of peritoneal dialysis patients experienced abnormal digestive symptoms such as acid reflux, nausea and vomiting, early satiety, and postprandial bloating, leading to poor appetite and malnutrition in peritoneal dialysis patients. Medications such as acid suppressants and gastroprokinetics are frequently used in Western medicine, but the long-term efficacy is unfavorable. It has been shown [7] that traditional Chinese medicine (TCM) provides significant efficacy in the treatment of gastrointestinal dysfunction in peritoneal dialysis patients with fewer adverse effects. It was found that spleen deficiency is the main type of evidence in ESRD patients, and blood stasis and dampness are present throughout the disease. Patients with ESRD have a depleted kidney essence and require care to protect kidney qi to replenish the innate kidney essence [8].

The development of coronary heart disease is linked to systemic atherosclerosis. Patients with elevated levels of medial calcification may provide insight into this phenomenon, so it is feasible to assess the hypothesis of death and prognosis of patients [9–11]. Thus, accurate determination of the degree of AS in patients or exploration of related biomarkers is of great importance for patient prognosis [12]. Previous approaches for the detection of arterial elasticity included central aortic pressure (CAP), CT, ultrasound, and X-ray plain scanning, but all of them exhibit limitations. In recent years, arterial pulse wave velocity (PWV) has been widely used in the detection of arterial elasticity and achieved certain clinical results [13, 14]. It contributes to the early identification and prevention of vascular sclerotic illnesses by identifying arterial elasticity, vascular stiffness, and vascular stenosis [15, 16].

It has been found that dialysate calcium concentration is one of the important factors affecting calcium homeostasis in patients on maintenance hemodialysis, and dialysate higher than blood calcium concentration increases the risk of disorders of calcium and phosphorus metabolism in patients, leading to a variety of complications [17]. In peritoneal dialysis, the mode of calcium ion transport through the peritoneum in dialysate varies from that in maintenance hemodialysis, and the possibility that dialysate calcium concentration still yields a greater impact on calcium and phosphorus metabolism and bone metabolism in peritoneal dialysis patients deserves further in-depth study. To this end, this study investigated the incidence of cardiovascular events in individuals with typical Parkinson's disease and documented alterations in serum sclerostin levels to evaluate the association between SO level and arterial stiffness in PD patients.

## 2. Materials and Methods

### 2.1. Research Subjects

50 patients with PD on continuous ambulatory peritoneal dialysis (CAPD) for more than 6 months in the nephrology department of our hospital were included in the study.

Inclusion criteria were as follows: (1) patients meeting the criteria for dialysis in the Clinical Guidelines for Hemodialysis [18]; (2) duration of dialysis ≥3 months; (3) aged >18 years; (4) with complete data; (5) with regular PD ≥ 3 months; and (6) with acute physiological and chronic health status II scores [19] <25.

Exclusion criteria were as follows:(1) patients with mental illness or mobility difficulties that prevented cooperation with the study; (2) patients who used hormones or immunosuppressants within the past one year; (3) patients who underwent surgery or had trauma within the past one month; (4) patient with other serious diseases, such as malignant tumors; (5) patients with mental illnesses such as dementia and impaired consciousness; (6) patients with immune system disorders; (7) patients with severe liver function and cardiac insufficiency; (8) patients during pregnancy; (9) patients who revoked their consent or died; and (10) patients with renal failure requiring renal transplantation treatment. This study was approved by ethics committee of Shexian Hospital of Traditional Chinese Medicine, No.8293799/1, and our patients and their families signed informed consent.

### 2.2. Methods

1. Collection of baseline patient profile, including age, gender, height, weight, BMI, smoking history, dialysis age, urea clearance index (Kt/V), residual renal function (RRF), diabetes mellitus (DM), diastolic blood pressure (DBP), and systolic blood pressure(SBP).
2. Biochemical indicators, including hemoglobin (Hb), albumin (ALB), total cholesterol (TC), urea nitrogen (BUN), creatinine (CREA), triglyceride (TG), uric acid (UA), parathyroid hormone (PTH), blood phosphorus (P), fasting blood glucose (GLU), corrective calcium (Ca), calcium-phosphorus product, low-density lipoprotein (LDL-C), and high-density lipoprotein (HDL-C), were recorded.
3. Detection of serum sclerostin concentration: the detection was performed with enzyme-linked immunosorbent assay (ELISA) double antibody sandwich method. 5 mL of fasting venous blood was collected from enrolled patients, and the supernatant was centrifuged and stored for testing. The levels of Hb, ALB, TC, BUN, CREA, TG, UA, PTH, GLU, Ca, LDL-C, HDL-C, BUN, P, Ca, and calcium and phosphorus were determined using a CX9 large automatic biochemical analyzer manufactured by Beckman Coulter, USA. The reagent kit was purchased from Tianjin Asil Biotechnology Co.
4. Determination of arterial stiffness: each patient was given an arteriosclerosis detector to record their vascular stiffness measurement (baPWV). Without taking age into account, arterial stiffness (BaPWV) of 1400 cm/s was considered a cutoff value, with a value below 1400 cm/s considered normal. The mild elevation is defined as 20–30% over the usual value, moderate elevation is defined as 30%–50% above the normal value, and severe elevation is defined as more than 50% above the normal value.

### 2.3. Statistical Analysis

SPSS 24.0 was used for data processing in this study. The counting data and measurement data were analyzed using the chi-square (X^2^) test and the *t*-test, respectively. Pearson linear correlation analysis was used for correlation analysis between data. *P* < 0.05 indicates a statistically significant difference.

## 3. Results

### 3.1. Comparison of General Data of Patients in Two Groups

Without regard for age, the eligible patients were assigned to a low PWV group and a high PWV group with brachial-ankle pulse wave velocity (Ba PWV) of 1400 cm/s as the cutoff value. Statistical significance was absent in patient characteristics despite more males in the high PWV group (*P*=0.055). The low PWV group had significantly lower mean age, SBP, SO, and PWV levels, fewer diabetic patients, and higher CREA than the control group (Table 1).

### 3.2. Analysis of PWV-Related Factors

PWV was shown to be correlated with age, SBP, PTH, P, Ca, GLU, and serum sclerostin while negatively correlated with CREA (Table 2).

### 3.3. PWV Multiple Regression Analysis

Multiple stepwise regression analysis showed that age, SO, and SBP demonstrated great potential to predict PWV (*P* < 0.05) (Table 3).

## 4. Discussion

With the increasing incidence of chronic kidney disease, more than 100 million people in China are suffering from chronic kidney disease, and a significant proportion of these patients have progressed to the end stage and require renal replacement therapy. Peritoneal dialysis is the main alternative therapy for patients with end-stage renal disease in China due to its simple operation, no site restrictions, and its advantages over hemodialysis in protecting patients' residual renal function and maintaining hemodynamic stability [20–22]. With the increase in the number of patients on peritoneal dialysis and the prolongation of patients' dialysis, patients' quality of life and dialysis efficacy have gradually been highlighted, and the factors affecting patients' quality of life and dialysis efficacy mainly include residual renal function, nutritional status, peritonitis, peritoneal function, and other related complications [23]. Many clinical studies have confirmed [24, 25] that TCM carries great significance in the prevention and treatment of dialysis-related complications in peritoneal dialysis patients and in improving the efficacy of treatment. ESRD belongs to the category of “edema” and “deficiency labor” in TCM, and spleen deficiency is considered the main type of evidence in ESRD patients, and blood stasis and dampness are present throughout the disease. Patients with ESRD have a depleted kidney essence and require care to protect kidney qi to replenish the innate kidney essence [26].

Sclerostin, a glycoprotein expressed by the SOST gene in osteocytes, is a newly identified protein implicated in bone-vascular axis metabolism and is hypothesized to be related to the development of arteriosclerosis and vascular calcification [27]. Sclerostin is a newly identified protein that regulates vascular calcification and has been found in calcified vascular smooth muscle cells in addition to bone-derived sclerostin [28, 29]. Studies have shown that serum sclerostin levels gradually increase with the progression of CKD, and the relevant mechanism is unclear [30, 31]. Increased cardiovascular and cerebrovascular events in patients with chronic kidney disease (CKD) may be associated with arteriosclerosis, and PWV, as an index of arterial stiffness, contributes to non-invasively diagnosing the severity of vascular sclerosis [32, 33]. Studies have shown that baPWV is a strong predictor of cardiovascular mortality in HD patients, and SO level may serve as a potential biomarker of atherosclerosis, whereas there is a dearth of relevant research. At present, non-invasive methods for PWV measurement based on waveform analysis include brachial-ankle pulse wave velocity (baPWV), heart rate, and multi-neck pulse wave (cfPWV), among which cfPWV directly reflects the degree of aortic stiffness and shows excellent clinical relevance. It is currently considered the gold standard for assessing aortic stiffness and cardiovascular events [34, 35]. Recent research has shown that hyperphosphatemia, high calcium-phosphorus product, and hyperparathyroidism could lead to vascular calcification, increased arterial stiffness, and an increased risk of cardiovascular events [36].

The analysis of PWV-related factors in the present study showed that PWV was positively correlated with age, SBP, PTH, SO, P, Ca, and GLU while negatively related with CREA. The results of multiple stepwise regression analysis indicated that the age, SBP, and SO were predictors of PWV (*P* < 0.05). SO level in PD patients is significantly related with vascular sclerosis severity, which provides a theoretical basis for the evaluation of cardiovascular disease in PD patients. The level of PWV in PD patients was correlated with age, BNP, brachial artery systolic blood pressure, Hb, and previous history of DM. It is indicated that the control of blood pressure, volume, and blood glucose is key to achieve vascular function protection.

This may be related to the small sample size of this study and possibly because this study did not group patients with or without other preexisting diseases. It has been suggested that hemodialysis corrects disorders of calcium and phosphorus metabolism, improves vascular calcification and arterial stiffness, and delays or blocks arterial calcification and sclerosis in patients with abnormal parathyroid function [37]. Active vitamin D deficiency is prevalent in peritoneal dialysis patients. Krause et al. [38] found that 58.8% of maintenance hemodialysis patients had 25-hydroxyvitamin D deficiency and that vitamin D deficiency increased mortality. Therefore, specific correlations are required in animal experiments.

The degree of vascular sclerosis is highly correlated with SO level in Parkinson's disease patients, which might provide a theoretical basis for the evaluation of cardiovascular illness in Parkinson's disease patients. High serum sclerostin level is a risk factor for deteriorated arterial stiffness. Given the limited sample size, the relevant results require further validation by expanding the sample size.

## Figures and Tables

**Table 1:** Comparison of general data of patients in two groups.

Factor	Low PWV group(*n* = 25)	High PWV group (*n* = 25)	*P*
Age	56.23 ± 13.24	65.43 ± 8.81	<0.001
Gender (male/female)	9/16	12/13	0.055
Height	158.01 ± 7.73	161.37 ± 7.49	0.314
Weight	59.38 ± 11.26	60.47 ± 10.63	0.658
BMI	23.57 ± 4.49	23.90 ± 3.61	0.621
Smoking	14	17	1.233
Dialysis time	30.31 ± 26.17	24.47 ± 15.31	0.131
Urea clearance index (Kt/V)	1.55 ± 0.54	1.67 ± 0.75	0.762
Residual renal function (RRF)	0.57 ± 0.63	0.59 ± 0.62	0.652
Systolic blood pressure (SBP)	134.34 ± 22.45	158.72 ± 22.36	0.006
Diastolic blood pressure (DBP)	83.76 ± 13.84	83.51 ± 14.27	0.112
Diabetes mellitus	2	8	<0.001
Hemoglobin (Hb)	114.67 ± 21.51	116.53 ± 18.74	0.591
Albumin (ALB)	37.39 ± 4.28	36.27 ± 3.64	0.138
Blood urea nitrogen (BUN)	23.15 ± 5.53	21.16 ± 5.62	0.145
Creatinine (CREA)	881.33 ± 247.83	742.41 ± 272.63	0.003
Uric acid (UA)	383.25 ± 93.69	404.92 ± 91.31	0.225
Parathyroid hormone (PTH)	2.09 ± 0.51	1.95 ± 0.49	0.775
Serum phosphorus (P)	1.66 ± 0.37	1.57 ± 0.35	0.104
Corrected calcium (Ca)	2.23 ± 0.32	2.21 ± 0.27	0.846
Calcium-phosphorus product	3.42 ± 1.43	3.38 ± 1.27	0.936
Total cholesterol (TC)	4.68 ± 1.02	5.03 ± 1.25	0.232
Triglyceride (TG)	2.03 ± 1.26	2.09 ± 1.28	0.832
Low-density lipoprotein (LDL-C)	3.15 ± 0.73	1.46 ± 0.97	0.42
High-density lipoprotein (HDL-C)	1.33 ± 0.35	1.44 ± 0.93	0.547
Fasting blood sugar (GLU)	5.63 ± 1.67	6.37 ± 2.56	0.083
Serum sclerostin	202.13 ± 20.14	433.37 ± 24.52	0.004
PWV	9.66 ± 1.35	13.36 ± 1.48	<0.001

**Table 2:** Analysis of PWV-related factors.

Factor	r	*P*
Age	0.428	<0.001
Dialysis time	0.096	0.274
Systolic blood pressure (SBP)	0.561	<0.001
Diastolic blood pressure (DBP)	0.026	0.761
Hemoglobin (Hb)	0.076	0.410
Albumin (ALB)	−0.142	0.102
Creatinine (CREA)	−0457	0.021
Parathyroid hormone (PTH)	0.662	<0.001
Serum phosphorus (P)	0.589	0.021
Corrected calcium (Ca)	−0.503	<0.001
Total cholesterol (TC)	0.112	0.378
Triglyceride (TG)	−0.101	0.441
Low-density lipoprotein (LDL-C)	0.006	0.952
High-density lipoprotein (HDL-C)	0.057	0.671
Fasting blood sugar (GLU)	0.238	0.027
Serum sclerostin	0.219	<0.001

**Table 3:** PWV multiple regression analysis.

Factor	*β*	*t*	*P*
Age	0.067	4.891	<0.001
Systolic blood pressure (SBP)	0.029	7.537	<0.001
Serum sclerostin	2.721	13.562	0.003

## Data Availability

No data were used to support this study.
